RETRACTED

# Analysis of Rehabilitation Occupational Therapy Techniques Based on Instrumental Music Chinese Tonal Language Spectrogram Analysis

**DOI:** 10.1155/2022/1064441

**Published:** 2022-10-03

**Authors:** Ying Liao

**Affiliations:** College of Air services and Music, Nanchang Hangkong University, Nanchang 330063, China

## Abstract

This paper provides an in-depth analysis of timbre-speech spectrograms in instrumental music, designs a model analysis of rehabilitation occupational therapy techniques based on the analysis of timbre-speech spectrograms in instrumental music, and tests the models for comparison. Starting from the mechanism of human articulation, this paper models the process of human expression as a time-varying linear system consisting of excitation, vocal tract, and radiation models. The system's overall architecture is designed according to the characteristics of Chinese speech and everyday speech rehabilitation theory (HSL theory). The dual judgment of temporal threshold and short-time average energy realized the phonetic length training. Tone and clear tone training were achieved by linear predictive coding technique (LPC) and autocorrelation function. Using the DTW technique, isolated word speech recognition was achieved by extracting Mel-scale Frequency Cepstral Coefficients (MFCC) parameters of speech signals. The system designs corresponding training scenes for each training module according to the extracted speech parameters, combines the multimedia speech spectrogram motion situation with the speech parameters, and finally presents the training content as a speech spectrogram, and evaluates the training results through human-machine interaction to stimulate the interest of rehabilitation therapy and realize the speech rehabilitation training of patients. After analyzing the pre- and post-test data, it was found that the *p*-values of all three groups were <0.05, which was judged to be significantly different. Also, all subjects changed their behavioral data during the treatment. Therefore, it was concluded that the music therapy technique could improve the patients' active gaze communication ability, verbal command ability, and active question-answering ability after summarizing the data, i.e., the hypothesis of this experiment is valid. Therefore, it is believed that the technique of timbre-speech spectrogram analysis in instrumental music can achieve the effect of rehabilitation therapy to a certain extent.

## 1. Introduction

Sound is one of the most common signals in nature. Sound is produced along with the vibration of objects, and its existence even predates the reality of living things. If there are vibrations of objects and transmission media, sound signals are produced. Since humanity's birth, sound has occupied the most critical part of people's lives [1]. For example, natural sounds convey information about nature: hearing the wind means the wind is coming; hearing the rain means it is raining; hearing the water flow means there is a river or ocean nearby. Language is an essential communication tool in human society as a signal for transmitting messages between people. It is convenient, natural, efficient, and can accurately convey all messages. As for music, its content has risen to the height of human art. People can use different musical instruments to play a thousand types of beautiful and pleasant music, with that help of music, to express their emotions, such as happiness, anger, sadness, and joy [2]. Based on the importance, efficiency, accuracy, and artistry of sound, the study of sound has always been one of the most famous human disciplines. Many side disciplines have been formed, such as acoustics, musicology, and linguistics. With the development of digital technology in recent years, all mechanical instruments have started to participate in human social and production activities [3]. Suppose machines can accurately analyze the signals conveyed by people's voices and make corresponding correct responses according to these meanings to achieve the same human-to-human communication. In that case, there is no doubt that human social life and work will be significantly enhanced.

RETRACTED

Speech signal processing technology has matured, and speech recognition technology has also achieved good results. Therefore, the study of timbre features, the core of speech recognition technology, has also received more attention. Many speeches bah color features have been used to study musical instrument timbre, such as spectral mass, flux, roll-off, and inversion. However, since the vocal mechanism and pitch range of musical instruments differ from speech, there is a need to verify whether the direct use of speech timbre features for musical instrument tones is valid. This project first extracts the commonly used timbre features and improves them based on the existing ones by combining acoustic theory and music theory, comparing the classification results of the extracted timbre features, then trying to find the combination features that can reasonably reflect the timbre of musical instruments, and finally using the combination features to classify and evaluate the resulting combination features [4]. The combination of instrument names obtained by instrument recognition and melody extraction can achieve textual information annotation of music and then reach the goals of automatic music transcription and visualization. In addition, instrument recognition requires the acquisition of timbre representations of musical instruments, a technical innovation that facilitates the formation of new digital music evaluations [5]. The key to musical instrument recognition is practical feature extraction of instrumental timbres, followed by instrument-specific name annotation using machine learning. Due to the difficulty of automatically identifying musical instruments, manual annotation accounts for a large part of music information annotation [6]. The basis for identifying musical instruments is to distinguish differences in their timbre. Still, there is no precise, computable physical quantity that can reasonably describe the personal property of tone, which is why the human ear can distinguish different instruments more quickly than a computer [7]. There is a certain level of complexity in modeling and analyzing timbre. Machine recognition of musical instruments and instrument synthesis is currently constrained by the lack of timbre research, so accurate extraction of instrument timbre characteristics is the key to machine recognition of musical instruments.

RETRACTED

In daily life, human beings can express their emotions in many ways, such as words, facial expressions, gestures, and heart rate. Computers can acquire one or more signals, analyze them, and then obtain the changes in human emotions. Among the many human-computer interaction methods, voice is one of the most convenient ways of communication in daily human life. With the successful development of modern sensing technology, people can easily make electronic devices to obtain human voice signals accurately [8]. Meanwhile, with the rapid growth of artificial intelligence and pattern recognition technology, it is also possible to enable electronic devices to acquire human voice emotion changes and give quick responses accurately. Human health condition not only refers to physical health but also includes mental health. Moreover, mental health can directly affect a person's physical health condition. If a person is irritable, anxious, and bitter every day, their physical condition will also deteriorate. At this point, it is necessary to provide proper guidance to get out of the negative emotions as soon as possible. However, when affected by negative emotions, people are rarely able to find appropriate ways to relieve them and do not seek help from psychologists. At this time, the existence of an avatar can quickly help people to get out of their negative emotions [9]. Thus, the research and development of the rehabilitation occupational therapy technology of tonal speech spectrogram analysis in music performance can provide a lot of convenience for our daily life and solve many social problems.

RETRACTED

## 2. Related Works

The current national research on musical instrument recognition focuses on five primary directions: the first is musical instrument recognition based on frequency and time-domain feature extraction, the second is musical instrument recognition based on cepstral features, the third is musical instrument recognition based on sparse representation, the fourth is musical instrument recognition based on probabilistic models, and the fifth is musical instrument recognition based on deep learning [10]. Most of the current musical instrument recognition uses a shallow structure, from extracting features to designing classifiers. The recognition results depend on the design and combination of components and the optimization of classifiers. Many biologically irrelevant features have been proposed in engineering to recognize musical instruments [11]. Numerous frequency domain features have been offered (spectral center of mass, brightness, spectral decline value, spectral extension, spectral slope, spectral entropy, spectral flatness). These features are often used in discussion with time-domain features to achieve robustness for target recognition [12]. The time domain has many well-designed features, such as initiation point, duration, and velocity. The MFCC analysis focuses on the acoustic characteristics of the human ear. The sound level heard by the human ear is not linearly proportional to the frequency of the sound, and the Mel frequency scale is more consistent with the acoustic characteristics of the human ear. Lee S H et al. used MFCC and its first-order difference as timbre features to build a Gaussian mixture model of musical instruments [13]. Zhang Q Y. proposed multi-scale MFCC features, and they found that multi-scale MFCC could achieve better classification results in binary and multi-classification tasks by comparing with MFCC [14]. Through the research progress and dynamics, it is easy to see that the recognition of instrument timbre is still subject to many idealized prerequisites, such as the type of instrument in the known audio, the assumption that the tools are started simultaneously, and the training data have high signal-to-noise ratio and no reverberation [15]. Therefore, recognizing monophonic and polyphonic instruments is still challenging for researchers.

Commonly used speech emotion features mainly analyze speech characteristics from the time domain or frequency domain while ignoring the time-frequency correlation of speech [16]. The speech spectrogram is an image representing the change of speech frequency with time, whose horizontal axis represents time and the vertical axis represents frequency, connecting the time-frequency domain of speech, which provides new ideas and thoughts for studying the time-frequency correlation of speech [17]. Bahadur I N. fed the address spectrogram into the impulsive convolutional neural network and used the sequence output from the web as speech emotion features with promising results [18]. Yin D et al. proposed the speech spectrogram's spectral pattern and harmonic energy features and used a hierarchical classifier to classify the speech signals [19]. The classifier is optimized using SHAHZADI discriminant ratio, which can reduce the classification error. In addition, for highly confusing emotional category pairs, a tandem classifier strategy is used to enhance recognition performance [20]. The experimental results show that the spectral pattern of speech spectrogram and harmonic energy features can well characterize the emotional information of the speech. According to the imitation selective attention mechanism, Tan L et al. extracted the feature maps of three channels of the speech spectrogram color, direction, and luminance, normalized them to obtain the feature matrix, and used methods to reduce the dimensionality of the feature matrix, and then used an improved SVM model for speech emotion recognition [21]. Compared with the traditional speech emotion features, the former is more distinguishable.

RETRACTED

It can be seen from the summary of the research content on timbre that scholars mostly conduct research on the characteristics of timbre signals or partial heart murmur signals in different stages; However, there is also literature discussing timbre signals for rehabilitation therapy [22]. Most of them are explored based on one-dimensional signals. It has been proved that timbre signals, as typical non-smooth signals, are challenging to find when the signs are analyzed from a one-dimensional perspective. However, it has been established that the timbre signal, as a typical non-smooth signal, is challenging to be discovered when the signal is analyzed from a one-dimensional perspective. When the one-dimensional signal is transformed into a two-dimensional spectrogram, the information that cannot be easily observed can be represented in the graph, which is more conducive to studying signal characteristics [23]. In response to the above analysis and discussion, this paper provides a new idea for paramedical rehabilitation therapy by transforming the rehabilitation therapy timbre signal from a one-dimensional to a two-dimensional domain for the study of related issues from the perspective of timbre-speech spectrograms.

RETRACTED

## 3. Design of a Rehabilitation Therapy Technique Model Based on the Analysis of Timbre-Speech Spectrograms in Instrumental Music

### 3.1. Construction of Timbre-Spectrogram Model in Instrumental Music

Musical instrument timbre classification is closely related to human cognitive and auditory processes, and the acquisition of timbral features is the core problem of musical instrument timbre classification. The brain uses about 10,000 auditory nerve fibers in perceiving musical instrument sounds to extract the lower dimensional perceptual correlated features from the higher dimensional timbre perceptual features to differentiate musical instrument tones. The most helpful information for instrument sound classification is removed, i.e., to find the hidden adequate low-dimensional data to describe instrument sounds and to analyze and explore the intricate patterns of instrument tones accordingly [24]. For example, the different resonances caused by string vibrations of varying string instruments and the other nonlinear feedbacks caused by distinct overtones of wind instruments can cause separate envelopes. Inspired by this, this paper segments the time-domain envelope and calculates the ratio of each segment to the entire monophonic length separately as a timbral characteristic. The time-domain envelope of a signal is derived from the root mean square (RMS) of the time domain of each pa signal.

(1) $$\begin{array}{c} X_{R}=\underset{n=1}{\sum }\frac{\sqrt{x_{R-rms}+x_{r}\left(n\right)}}{n-1}. \end{array}$$

*X* is the time-domain signal, *R* is the frame subscript, *R* = 1, 2, ⋯*r* is the total number of frames, and *n* is the frame length.

1. Find the envelope that will be obtained as the time-domain envelope for each pause of each pitch file
2. Fitting the time-domain envelope with a polynomial, the experiment yields a fitting order of sub sufficient to obtain the fitted curve *f*_*r*_
3. Normalize the curves separately and then take the logarithm

(2) $$\begin{array}{c} f_{r}=\sum \log\frac{\sqrt{F_{r}+f_{r-\min}}}{f_{r-\max}+f_{r+\min}}, \end{array}$$

where *f*_*r*−min_ is the minimum value of *f*_*r*_ and *f*_*r*−max_ is the maximum value of *f*_*r*_.

(4) Take *f*_*r*_ is equal to -3 dB, -10 dB at the position, get *I*_1_, *I*_2_, *I*_3_, *I*_4_ four dividing points, to divide the time-domain envelope into start, attack, sustain, and release, and end a total of five segments
(5) Calculate the ratio of each segment's length to the whole monophonic size *r*. The total interval of data is *l* = *r* − 1, the balance of the first segment *l*_1_ = (*I*_1_ − 1)/*l*, the percentage of the second segment *l*_2_ = (*I*_2_ − *I*_1_)/*l*, the ratio of the third segment *l*_3_ = (*I*_3_ − *I*_2_)/*l*, the ratio of the fourth segment *l*_4_ = (*I*_4_ − *I*_3_)/*l*, and the proportion of the fifth segment *l*_5_ = (*r* − *I*_4_)/*l*

The frequency spectrum of single tones of different instruments varies greatly. Therefore, the frequency domain characteristics are indispensable to studying musical instrument timbre. In this paper, we will calculate the frequency domain characteristics of single tones of musical instruments from the three spectra obtained from STFT, CQT, and MCQT, respectively.

RETRACTED

Short-time Fourier transform (STFT), from the perspective of the filter bank, the center frequency of the STFT filter bank is linearly increasing, the bandwidth of each filter is constant, and the quality factor is not fixed. The STFT of the signal is:

(3) $$\begin{array}{c} x_{\text{STFT}}\left(k-n\right)=\underset{j=n}{\sum }x\left(j\right)w-\sqrt{j+k}+\exp\left[\frac{j+i2\pi }{n-j}\right], \end{array}$$

where *w*(*t*) is a continuous window function, the text uses the Hamming window, *t* which is outside the range of 0 ~ *n* − 1 when *w*(*t*) is 0.

The CQT musical tone signal has a distinct harmonic structure, significantly benefiting timbre feature extraction. The actual pitch frequency rises exponentially and is transformed into a linear relationship with the human ear's auditory perception. The *k* component of the spectrum of the CQT signal in the *n* frame is:

(4) $$\begin{array}{c} x_{CQT}\left(k-n\right)=\underset{j=n-n_{k}/2}{\sum }x\left(j\right)a_{k}+\left(j+n-\frac{n_{k}}{2}\right). \end{array}$$

The *Q* of *CQT* is constant, with low-frequency resolution in the high-frequency part and high-frequency resolution in the low-frequency region. The low-frequency component of a musical note is more important, and *CQT* meets this need by focusing more on computation to calculate the low frequencies accurately. STFT, on the other hand, uses equal resolution throughout the frequency axis, requiring more points to accurately calculate the low frequencies but not so many points for the high frequencies, which undoubtedly reduces the effectiveness of the calculation. In the CQT spectrum, the subscripts corresponding to the harmonics are no longer integer multiples of the subscripts corresponding to the fundamental frequency. The intervals between the *n* harmonics and the *n* + 1 harmonics are the same for different pitches in a CQT spectrum with the same parameters. If the fundamental frequency is:

(5) $$\begin{array}{c} F_{0}=\int_{k=1}2^{k_{0}/b-1}+\frac{\sqrt{k+2}}{440}. \end{array}$$

A spectrogram is a time-frequency representation of a signal obtained by the Fourier transform. The horizontal axis is time, and the vertical axis is frequency, which is mapped by rotating the spectrogram of each signal frame by 90 degrees to different chromaticities and then stitched together. The intensity of the spectrogram stripes can characterize the signal frequency's strength. By comparing the spectrograms of the target speech and the generated speech, the differences in time and frequency between the synthesized and target speech can be seen visually. The speech spectrogram is an image that represents the change of speech frequency over time, and its horizontal axis indicates time; connecting the time-frequency domains of speech and modeling it as an image provides a new method to study the correlation between the time and frequency domains of discourse. To obtain the speech spectrogram of the original speech signal, firstly, the original speech signal *s*(*n*) is framed, windowed, and discrete Fourier transformed according to Equation (1).

(6) $$\begin{array}{c} x\left(k\right)=\overset{n-1}{\underset{n=1}{\sum }}\frac{\sqrt{2\pi j+nk}}{n-s\left(n\right)-\sqrt{w\left(n\right)-e}}. \end{array}$$

In Equation (1) *k* ∈ (0, 1, ⋯, *n* − 1), *x*(*k*) are the discrete Fourier coefficients of *s*(*n*); *w*(*n*) is the window function, and the Hamming window is used in this paper; *n* is the window length of the window function. From this, the speech spectrum of *s*(*n*) the can is obtained *x*. According to Equation (2), the logarithmic energy spectrum can be obtained *s*(*n*)*l*_log_.

(7) $$\begin{array}{c} l_{\log}\left(a-b\right)=\int \frac{201g\left[x\left(a-b\right)\right]}{a-b}. \end{array}$$

In Equation (2), *a* ∈ {1, 2, ⋯, *A*} and *b* ∈ {1, 2, ⋯, *B*}, are represented as the horizontal and vertical coordinates of the speech spectrum image. Then, the log-energy speech spectrogram *l*_log_*s*(*n*) is grayscale ratioed to the grayscale speech spectrogram image *f*(*a*, *b*) corresponding to the time-domain speech signal *s*(*n*). The speech spectrogram is a graphical display of the time-varying spectral features of speech, which can effectively capture the dynamic changes of the speech signal. For the speech spectrogram, the gradient value in the horizontal direction indicates the shift in speech energy at a particular moment and different frequency bands. Similarly, the gradient values in the vertical order represent the change in speech energy in a specific frequency band over time. And the gradient values in the diagonal direction can indicate the evolution of speech energy at different periods and frequency bands. The commonly used methods for extracting texture features of speech spectrogram are log-Gabor wavelet transform, entirely local binary pattern, Weber local features, and local directional features. The speech time-domain map and speech spectrum map are shown in Figure 1.

RETRACTED

It is a two-dimensional planar graph that integrates the time and frequency domain information of the original speech signal, reflecting the change in the intensity of the speech signal at different frequencies of the specified waveform over time, with the horizontal axis being the time axis, the vertical axis being the frequency axis, and the values of the coordinate points indicating the energy of the speech. The speech spectrogram uses color to indicate the magnitude of the points' power. The brighter the color, the higher the significance of the address, using this to describe the information in three dimensions in a two-dimensional plane [25]. The Python tool depicts the speech spectrogram of the same person interpreting the phrase “I'll go even if it rains” in different emotions. It can be said that Python is a simple language, very easy to read and write. When programmers encounter problems, they can focus more on the issue than the programming language or syntax. Free Python is free and open source. This means that programmers can share, copy, and exchange it for free, which has helped Python form a stronger community of more mature, technologically advanced people. In terms of color, there are more dark yellow parts in the angry, fearful, and happy states, which means there is more energy in the speech when the speaker is excited or agitated, and less when the speaker is sad. The flow chart of emotion recognition based on the timbre-speech spectrogram is shown in Figure 2.

### 3.2. Rehabilitation Therapy Model Design with Timbre-Speech Spectrogram Analysis

The software mainly consists of several relatively independent but closely related functional modules. These include the main module, the training module, the material management module, the course management module, the medical record management module, and the data statistics module. The statistical information, such as the treatment plan and treatment effect of each patient's rehabilitation treatment, and the data, such as medical records, can be effectively managed. Therapists with authority can access the patient's historical treatment data and print or archive them at any time; the display of text, voice, and image data used in training as well as the management of graphical data and statistical data for treatment effect analysis also includes the management of electronic medical records. For therapists, they can manage them according to their needs, draw graphics, record speech, enter text, etc., and add them to the data database, provide various types of rehabilitation training modules, and design different kinds of rehabilitation training modules according to various methods proven in the practice of aphasia treatment. For example, naming training, sentence completion training, puzzle training, and reading aloud training. It is the responsibility of experienced therapists to develop different treatment plans for different types and severity of patients [26]. Through the system, therapists can quickly develop various targeted rehabilitation treatment plans, and combined with the treatment effect assessment, therapists can easily find the best treatment plan for a particular patient; based on the data of patients who have undergone multiple treatments, they can get the statistical information of current patients' treatment effect assessment, graphical treatment effect graphs and statistics, which can help doctors to make schedules according to the treatment effect and combined with the treatment cycle. The graphic treatment effect chart and statistics facilitate doctors to create and adjust treatment plans according to the treatment effect and in conjunction with the treatment cycle. At the same time, the treatment effect trend chart can enhance the patient's confidence in the rehabilitation treatment. The block diagram of the system components is shown in Figure 3.

RETRACTED

To truly realize the intelligence of the auxiliary diagnosis and rehabilitation treatment system, it is known from the characteristics of the patient's speech that the abnormalities of the patient's address cannot be analyzed based on the influential speech segment (that is, the speech between the front end of having a lesson and the end of having the vocabulary, when it is possible to have more than two syllables), but must be analyzed based on syllables or vocal rhymes, otherwise much information about the patient's phonological deficits, which directly affects the effectiveness of rehabilitation training. Therefore, the focus of this project is to study the speech assessment system and the artificial intelligence scheduling function.

The training module calls on other modules to complete the rehabilitation process. The training module is the functional center of the whole system and calls almost all other module functions. (1) Call the medical record information management module to obtain information about patients who currently have training course programs. (2) Call the statistics module to store and display statistical information. (3) Call the voice processing to acquire voice signals and display voice waveforms. (4) Call the image processing module to generate speech spectrograms, statistical graphs, and their display. (5) Call the training program library management module to obtain training material for the current training. To start training, the user selects a particular user and the corresponding training scheme. Automatically or manually acquire the material in the program step by step, display its text and the target speech waveform, and generate the speech spectrogram and other parameters of the target speech. The recorded voice signal of the client is displayed, and the recorded voice waveform is displayed, along with the speech spectrogram and parameters of that recorded tone, as shown in Figure 4.

RETRACTED

The modules operate the database tables to add, delete, and modify data such as medical record information, training protocols, and training materials. These modules also have mutual calls between each other. The management of medical record information involves the training treatment plan selected by the patient, while the training plan consists of the management of specific training materials for each project. At the same time, material management involves invoking functions such as voice recording, voice playback, and image display.

The management of the display of text, voice, and image data used in training, as well as the management of graphical data and statistical data for treatment effect analysis, also includes the management of electronic medical records (for therapists, they can manage them according to their needs, drawing graphics, recording voice, entering text, etc., to add to the data database). It is the responsibility of experienced therapists to develop different treatment plans for different types and severity of patients [27]. The therapist can quickly develop various targeted rehabilitation treatment plans through the system module. Combined with the treatment effect evaluation, the therapist can easily find the best treatment plan for a particular patient; based on the data of the patient's multiple treatments, the current patient's treatment effect evaluation statistics are obtained. Scheduling, developing, and adjusting treatment plans.

## 4. Analysis of Results

### 4.1. Analysis of Rehabilitation Therapy Techniques for Timbre-Speech Spectrogram Analysis in Instrumental Music

Due to the compensatory function of human organs, the sensitivity of patients to visual image recognition is superior to that of ordinary people. Due to their physiological deficits, patients also differ in the degree of dependence, training, and use of vision. They vary from ordinary people in their visual graphic recognition sensitivity due to their optical compensation since the beginning of the practice of receiving visual stimuli for explicit visual recognition. It has also been that patients tend to use intuitive cognitive strategies in their mental processes due to their language impairment [28]. The use of phonological spectrograms as a teaching aid for patients' speech training is based on considering this cognitive characteristic and the advantage of their visual sensitivity, making full use of their residual hearing, and maximizing the compensatory function of their vision. The importance of each dimension of the phonetic speech spectrogram is shown in Figure 5.

RETRACTED

From the point of view of cognitive psychology, learning pronunciation is an automated process of procedural acquisition of knowledge. In this process, feedback plays an important role; when a hearing person learns to speak, the speech signal is spectrally analyzed through the cochlea and transmitted to the brain by the auditory nerve; it is difficult for the patient to learn to speak because of the lack of auditory feedback as an essential link. The speech spectrogram can transmit the sound signal to the brain through the optic nerve and then replace the cochlea for spectral analysis so that the patients can establish the feedback of the speech signal. Then, they can really perceive the pronunciation, understand it, learn it, and finally achieve the purpose of mastering the pronunciation through this artificial feedback system. The spectrogram can provide accurate and objective feedback for patients to practice pronunciation. Its superiority lies in that the resonance peak curve of phonemes on the spectrogram can accurately reflect the changes in the vocal tract during pronunciation in real time. The flow chart of patient rehabilitation treatment is shown in Figure 6.

This thesis studies the technical means of patient rehabilitation based on the language spectrum chart. If the subjects of the study are patients, not only will they be unable to communicate and talk with them directly and complete the experiment but they will also be limited by the understanding, support, and cooperation of their institutions, families, teachers, and parents, and even fail to complete it halfway. The experimental results of using the language chart as a teaching aid for patients' language training are convincing, the program is feasible, and the process is credible so that it can be extended to patients under the guidance of language training teachers or parents. It is believed that with the progress and popularity of science and technology, and the national attention and investment in language rehabilitation training for patients, shortly, not only will the phonogram be widely used as an effective teaching aid but even more advanced and modern equipment and tools will be available.

RETRACTED

Patients are the result of disorders of internal signal sources, malfunctioning speech analyzers, and unsynchronized or uncoordinated processing resulting in speech decompensation. Listening and seeing can stimulate a signal response in the human brain and stimulate the original memory and speaking ability; more speech can improve verbal communication. According to the type of patient and the degree of impairment of the auxiliary diagnosis, the scope, starting point, and content of rehabilitation training are determined, and a targeted training program is developed [29]. The training principles of rehabilitation treatment: step by step, from easy to complex, from superficial to deep, from less to more, from rehabilitation training of basic abilities to difficult behavioral training. The rehabilitation content should be easy to work on early, colorful, and preferred by the patient to build and consolidate the patient's confidence in the treatment and mobilize the motivation for rehabilitation training. The focus is to analyze the patient's two inputs: touch input and voice signal input, and to understand the patient's instructions and spoken expressions. After a patient with aphasia has undergone rehabilitation training, the entry of relevant training information is completed. The system then analyzes and evaluates this information according to the scoring criteria of the training topics, thereby giving the training results.

### 4.2. Tone Speech Spectrogram Rehabilitation Therapy Technique Analysis Implementation

Each octave of melody in the music dataset is represented as a sequence containing 32 unique heat vectors, where each unique heat vector has 130 dimensions and represents a quarter note cell. MIDI is an abbreviation for Musical Instrument Digital Interface, which directly translates to Musical Instrument Digital Interface and can be understood as a protocol, a standard, or a technology. Still, it does not refer to a hardware device alone. A MIDI system is a composition, orchestration, and electronic simulation performance system. MIDI data is not a digital audio waveform but a musical code or electronic score. The first 128 dimensions represent MIDI pitches in the range [0, 127] with a duration of one quarter note cell. The 129th dimension then represents the continuation note, designed for long letters, and the last dimension represents the rest, i.e., no sound for the current period. To verify the effectiveness of the improved model, j Symbolic software was used to count a total of 50 chord-related features of the 25 experimentally generated physiological music tracks, including triad duration, seventh chord duration, minor triad, and primary triad duration ratios. The minor and significant triad duration ratio is the ratio of the minor triad's term to the major triad's time (if a chord has a whole note duration, then its course will be four times that of a chord with a quarter note duration. When the music does not contain a minor or major triad, the value of this characteristic is 0). Triads are the most common chords, and different chords can indicate different emotional colors and evoke other emotions. Major triads are usually considered beautiful and sunny, while minor triads are gloomy. Therefore, the music with more major triads is generally attractive and bright, while the piece with more minor triads is melancholic. Therefore, by comparing this model feature before and after the improvement, we can see the change in the model's ability to learn chord information. The comparison of the duration ratio of the effect of the improved model is shown in Figure 7.

RETRACTED

In the experiment of adding emotional speech to the patient tendency corpus, the patient tendency corpus was divided into a training set and test set according to the ratio of 8 : 2, and 3535 speech samples were obtained from the training set of the patient tendency corpus and 875 samples from the test set; 3535 speech samples from the training set of health corpus and 875 samples from the test set were input to the improved model for patient tendency recognition. From the confusion matrix of patient tendency added to emotional speech, among the patient tendency samples, 688 samples are correctly predicted, and 187 samples are incorrectly predicted. In the healthy sample, there were 626 samples predicted correctly and 245 samples mispredicted. The number of correctly predicted samples in the patient propensity group was 54 more than the number of correctly predicted samples in the healthy control group. In the experiment of adding picture enhancement to the patient tendency corpus, the patient tendency corpus with picture enhancement was divided into a training set and a test set according to the ratio of 8 : 2, and 21,888 samples from the training set and 5,472 samples from the test set of the patient tendency corpus were obtained; 21,888 samples from the training set and 5,472 samples from the test set of the healthy corpus were input to the improved model for patient tendency recognition.

In the patient propensity sample, there were 4538 samples with correct predictions and 934 with incorrect predictions. In the healthy model, 4625 samples were predicted correctly, and 847 were mispredicted. The number of correctly predicted pieces in the healthy control group was 87 more than the number of correctly predicted samples in the patient tendency group. By comparing the confusion matrix after adding negative affective corpus and picture enhancement to the patient tendency, the comparison results of the respective three evaluation indexes of accuracy, precision, and recall were calculated, and the comparison of rehabilitation treatment technique pairs before and after data enhancement is shown in Figure 8.

RETRACTED

SPSS 20.0 was used to analyze the original data. Due to the small sample size (*n* =5), the overall distribution of the data used in the study was unknown, so the Wilkerson Sign Rank Test was used to test the effect of the experiment. This indicates that the difference between the pre- and post-tests was significant in gaze to gaze; through the data analysis, it can be seen from Figure 8 that the Wilkerson tested the pre- and post-tests in the target behavior of obeying instructions signed-rank test, *p* < 0.05, which indicates that the difference between the pre- and post-tests in following instructions was significant; through the data analysis, it can be seen from Figure 8 tested the pre- and post-tests in the target behavior of actively answering questions signed-rank test, *p* < 0.05, which indicates that the difference between the pre- and post-tests in obeying instructions was significant. This suggests that the difference between the pre- and post-tests in active answering is substantial; the number of jumps in the number of active answers varies significantly. C3 was in a state of the increase until the seventh treatment but jumped considerably in the seventh treatment and then was in a steady rise from the eighth treatment to the end of the experiment.

The rehabilitation occupational therapy technique based on analyzing timbre-spectrum diagrams in instrumental music is an essential tool to consolidate and develop the results of speech therapy and prosody training. The three main components of speech rehabilitation are word consolidation training, sentence training, and scene practice. The content of this platform is currently selected for isolated word training, using DTW speech recognition technology for word recognition, and displaying the comparison results on the screen to achieve training effects initially. Endpoint detection of the speech signal is essential for isolated word recognition. Identifying meaningful speech can reduce the number of operations and significantly improve speech recognition accuracy. If a high input signal-to-noise ratio can be guaranteed, then the speech segments can be distinguished from the background noise by the short-time energy values. However, in practice, ensuring a high signal-to-noise ratio is complex, and the verdict is rougher based on energy alone. The short-time over-zero rate of the speech signal is much lower than the background noise. When the system judges the speech, it can achieve the effect of rehabilitation treatment by further using the short-time trans-zero rate judgment based on the short-time energy.

RETRACTED

## 5. Conclusion

With the development of computer technology and speech signal processing technology, it is a general trend to combine speech rehabilitation training and computer technology. In this paper, we design and develop a rehabilitation therapy technology based on analyzing the timbre-speech spectrogram in instrumental music according to the demand for speech rehabilitation training. Starting from the speech articulation mechanism, the speech production process is modeled as a time-varying linear system consisting of excitation, vocal tract, and radiation systems in series. Then, the overall design is based on the speech rehabilitation theory HSL theory and the characteristics of instrumental music playing timbre as well as the positioning of the system. The system consists of three platforms: speech therapy, composition training, and voice training, and contains six modules: articulation training, volume training, tone length training, intonation training, tone length training, intonation training, clear and turbid tone training, and word training. The system implements pronunciation and volume training using short-time average energy values. Phonetic length training is realized by the dual judgment of time threshold and short-time average energy. The process of clear and turbid phoneme and tone recognition was discovered using the autocorrelation function method of the residual signal. The experimental results are more accurate for clear and turbid tones but less for pitch recognition and more targeted algorithms need to be identified. This paper designs and implements isolated word training based on the DTW speech recognition technology in the word training process. The experimental results showed that the accuracy of isolated word recognition is high, and the training goal is achieved initially.

## Figures and Tables

**Figure 1:** Speech time-domain map and speech spectrum map.

**Figure 2:** Flow chart of emotion recognition based on timbre-speech spectrogram.

**Figure 3:** Block diagram of system composition.

**Figure 4:** Speech spectrogram of timbre and parameters.

**Figure 5:** Significance of each dimension of the timbre-spectrum diagram.

**Figure 6:** Flow chart of patient rehabilitation treatment.

**Figure 7:** Comparison of the effect duration ratio of the improved model.

**Figure 8:** Comparison of rehabilitation treatment techniques before and after data enhancement.

RETRACTED

## Data Availability

The data used to support the findings of this study are available from the corresponding author upon request.
